The article "Modelling Behaviour of a Carbon Epoxy Composite Exposed to Fire: Part II—Comparison with Experimental Results" was published in 2017. Journal: Materials (Basel).

# Modelling Behaviour of a Carbon Epoxy Composite Exposed to Fire: Part II—Comparison with Experimental Results

**DOI:** 10.3390/ma10050470

**Published:** 2017-04-28

**Authors:** Pauline Tranchard, Fabienne Samyn, Sophie Duquesne, Bruno Estèbe, Serge Bourbigot

**Affiliations:** 1 UMR 8207, Unité Matériaux et Transformations (UMET), University of Lille, Lille F 59 000, France; pauline.tranchard@univ-lille1.fr (P.T.); fabienne.samyn@ensc-lille.fe (F.S.); sophie.duquesne@ensc-lille.fr (S.D.); 2 Thermal Tech Centre, AIRBUS Operation S.A.S, 316 Route de Bayonne, Toulouse 31060, France; bruno.estebe@airbus.com

**Keywords:** finite element analysis (FEA), fire testing, carbon fibre reinforced epoxy laminates, anisotropy, delamination, surface interactions

## Abstract

Based on a phenomenological methodology, a three dimensional (3D) thermochemical model was developed to predict the temperature profile, the mass loss and the decomposition front of a carbon-reinforced epoxy composite laminate (T700/M21 composite) exposed to fire conditions. This 3D model takes into account the energy accumulation by the solid material, the anisotropic heat conduction, the thermal decomposition of the material, the gas mass flow into the composite, and the internal pressure. Thermophysical properties defined as temperature dependant properties were characterised using existing as well as innovative methodologies in order to use them as inputs into our physical model. The 3D thermochemical model accurately predicts the measured mass loss and observed decomposition front when the carbon fibre/epoxy composite is directly impacted by a propane flame. In short, the model shows its capability to predict the fire behaviour of a carbon fibre reinforced composite for fire safety engineering.

## 1. Introduction

In a virtual testing approach, the development of predictive tools of the thermophysical behaviour of composite exposed to fire is an ambitious objective and one that is very promising. It is important to fully understand how the material behaves before any modelling. A previous work on the fire behaviour of the T700 carbon fibre-reinforced M21 epoxy resin composite laminate has been done [1]. It fully described complex physical, thermal and chemical phenomena (thermal expansion inducing formation of cracks, thermal degradation of the resin, internal pressure phenomenon, gas migration through the material, and thermal delamination). All of these analyses provide crucial data to validate a methodology developed for modelling the behaviour of a composite laminate exposed to fire. This two-part paper reports on the modelling of the thermochemical behaviour of a carbon fibre reinforced epoxy laminate exposed to fire. In Part I, the temperature-dependant thermophysical properties of the T700/M21 composite were determined and will be used in Part II (the present study), which reports on a developed three-dimensional (3D) thermochemical model applied to a fire test.

This section reviews how authors model in practice the fire response of composite. The approach is to obtain a complete model that is split into four distinct parts: the thermophysical model, the flame model, the modelling of the interaction between the fire and the composite, and the thermo-mechanical model. These four models can then be coupled. In this study, we focus on the thermophysical model (ignoring the thermomechanical aspects) and including input parameters that have a real physical sense (no search of best-fitting parameters).

Since the 1980s, considerable progress has been made on the development of mathematical models. More sophisticated models have been developed to predict the thermal response of decomposing laminate exposed to a high temperature. Different phenomena were taken into account such as heat conduction, decomposition, strain, volatile and moisture flow, and char formation. Damages were also introduced in the models with temperature rise, extend of char formation, expansion, internal pressure, delamination and cracking [2,3,4,5,6,7,8,9]. However, these models can be more or less sophisticated and can potentially require many input parameters describing the material, namely its thermophysical properties such as heat capacity, thermal conductivity or density. Despite those developments, models are limited to simplified flat materials using a one or two dimensional approach. Moreover, they are not necessarily applicable for all types of materials.

In the last decade, a variety of models of behaviour of composite in fire has been developed. Mouritz et al. produced an interesting review in 2009 [9] applied to different composites (sandwich materials or laminates composed of phenolic, vinyl ester, balsa, glass fibres, carbon fibres, etc.). They reported that major advances in the structural modelling of composites are completed, but that further analysis and validation against experimental data are required. Finally, one of the main priorities is obtaining a comparison between experimental and numerical results and to clearly determine the inputs of models.

In the case of the carbon fibre/epoxy laminate composite, it was demonstrated that the thermal degradation of an epoxy resin is different from one system to another and that generalisation is difficult. Indeed, there was evidence that the thermal decomposition and fire behaviour of a carbon fibre reinforced epoxy depends on the chemical nature of the hardener, the epoxy monomer used and the type, content and orientation of the fibres used [10,11]. Thus, it is important to better understand how the material behaves before any modelling. Moreover, authors have demonstrated that a basic model is not sufficient to model its burnthrough fire behaviour [12,13,14,15]. In 2003, the Gibson et al. model predicted a burnthrough time of 8.9 min instead of 3.6 min, obtained experimentally on a carbon fibre/epoxy composite. Moreover, in 2011, Sikoutris et al. predicted only the first 40s temperature at the rear face of the carbon fibre/epoxy composite submitted to the ISO2685:(E) test [16]. Most recently, Tranchard and Thomas predicted the temperature profiles near the impacted face and only the first 30s of the rear face temperature of a carbon fibre/epoxy composite submitted to a burnthrough test following the FAR25.856(b):2003 [17]. To sum up, all the authors concluded that other phenomena had to be taken into account in the modelling of carbon fibre/epoxy in fire, such as the thermal delamination. According to these authors, the modelling of the carbon fibre/epoxy composite submitted to fire (flame impinging the material) or to a high radiative heat flux is complex because all of the phenomena influence each other and they have not been fully taken into account in the model.

Nevertheless, authors succeed in predicting the thermal response of carbon fibre reinforced epoxy composites in specific conditions when submitted to a controlled heat flux (as radiative heat flux or time/temperature curve). In the case of controlled heat fluxes applied on carbon fibre reinforced epoxy composite, the results of the numerical and experimental results align [18]. In 1991, Mike and Vizzini [19] predicted the rear temperature profile of a carbon fibre/epoxy exposed to a 17.6 kW/m² heat flux up to the apparition of the thermal delamination (after six minutes of exposure). They used a three dimensional (3D) thermal model taking into account the energy accumulated by the material and the anisotropic heat conduction. In the last decade, McGurn and Desjardin [20] developed a model based on the extensive property data provided by the study of Quintiere et al. [21]. A carbon fibre/epoxy composite was exposed to cone calorimeter tests at different heat fluxes (25, 50, 75 and 100 kW/m²). A fairly good agreement was found between the experimental and numerical Heat Release Rate (HRR) curves for the four heat flux conditions. The authors explained that this model captures the data qualitatively (i.e., it captures the double peak history of the HRR but not the measured value). The model includes the energy accumulation, the heat conduction, the thermal decomposition, and the volumetric swelling. The authors employed phase-averaging principles to determine the macroscopic structural response from the microscopic changes in the fibres and resin. For this carbon fibre/epoxy composite, the authors noticed the influence of the swelling phenomena on the HRR response. They explained that the discrepancies were due to three factors: (1) an uncertainty of the heated back boundary condition for the gas transport (closed or open); (2) the combustion of gas released from the decomposition are not taken into account in the boundary conditions at the impacted face; (3) the permeability model needs to be improved.

More recently, experiments are carried out by submitting a T700/M21 to a controlled radiative heat flux [11] (Mass Loss Cone Calorimeter test, MLCC–ISO13927 [22]). The experimental results were discussed and compared to a 3D model including energy accumulation by the material, heat conduction, thermal decomposition and gas transport through the material. A complete set of material properties and of well-defined boundary conditions have permitted experimenters to predict with a reasonable certainty the thermal response and mass loss of the T700/M21 at 50 kW/m² [11]. The authors have reported that the accuracy of the model depends upon the accuracy of the thermal transport properties, the kinetic properties and the boundary conditions. They have shown that modelling the fire using well-known boundary conditions is complex because of the interactions between the flame and the gas phase of the material.

The strength of these previous models is that the heat flux condition at the impacted face was totally controlled (as MLCC [22], furnace test with the temperature increase which follows an ISO834 curve [23]). Thus, if the heat fluxes at the impacted and non-impacted faces are known, it is possible to predict the behaviour of the composite, but it is more complicated in the case of the direct impact of the flame on the composite.

Sophisticated models are reported in the literature but some of them do not succeed to model the behaviour of the composites. The more sophisticated the model, the more input data that must be determined. It is therefore important to highlight that some authors compared their numerical results with their experimental results. They have shown quite good agreement between both whereas others authors did not validate the numerical results with data from experiments. In all the cases, the main issue is that the determination of the input data is not fully detailed and the physical sense can sometimes be lost by fitting experimental curves. The determination of the physical and thermal properties of materials seems to be the key to obtain a suitable physical model. In the frame, the development of methods to determine thermophysical parameters of the T700/M21 composite was reported in the first-part of the paper [24].

First, the behaviour of the T700/M21 composite was investigated when exposed to fire [1]. Then, all input data for the model were measured and fully explained [24]. Therefore, the purpose of this paper is to compare the experimental data from a fire test (i.e., the temperature profile and mass loss) to their respective numerical simulations.

## 2. Small-Scale Fire Test

A novel fire test was developed to investigate the thermophysical behaviour of the T700/M21 composite in fire (the complete details of the test is given in a previous work [1]). During a single test (Figure 1), both condensed and gas phases can be simultaneously studied measuring the temperature profile and the mass loss and studying the nature and quantity of volatile gaseous species. The propane-air flame characterised by a heat flux is compliant with heat fluxes of two aeronautical certification fire tests: ISO2685:1998 [16] and FAR25.856(b):2003 [17]. In this paper, the test consists of impacting a 150 × 150 mm² sample by a propane flame at 1100 °C and with a calibrated heat flux of 116 kW/m².

## 3. Choice of the 3D Model Used

The aim is to develop a 3D suitable model including physical sense as much as possible while minimizing the number of inputs. A phenomenological approach was thus followed. We know that complex phenomena occur but some assumptions have to be made. First, the moisture effect is neglected since the fire experiments and characterisations did not exhibit moisture absorption by the material. In the literature, some papers demonstrated that epoxy resin are sensitive to moisture [25], but others did not [26]. This assumption renders the model less sophisticated. Then, the assumption of thermal equilibrium between the gas phase and the solid phase is considered. Moreover, the ablation is not considered since the analysis of experimental tests shows that the front face temperature of the panel does not reach sufficient temperature leading to thermochemical ablation [1]. In addition, the goal is to get a thermochemical model and so, the structural effects like expansion/contraction, mechanical delamination and mechanical erosion are not taken into account here. One of the main assumptions is considering the volume of the material as constant. Finally, the developed model considers the heat transfer, the decomposition of the composite, the gas production and their transport into the material linked to the internal pressure. All these phenomena are expressed in the governing equations.

A numerical thermochemical model was developed to predict the temperature profile of materials, the weight change, the gas mass flow and the internal pressure of materials. It is actually integrated into the commercial software SAMCEF (V17.003, Siemens PLM Software, LMS Samtech Company, Liege, Belgium) by the Amaryllis module used for the convenience of the engineering application. The energy equation, the rate of decomposition, the continuity equation and Darcy’s law, which are implemented in SAMCEF, are presented below.

### 3.1. Decomposition of the Material

The determination of the kinetic decomposition model was performed in a previous work [11] and presented in the first-part of this paper [24]. It is a two-step decomposition model including an autocatalytic reaction being competitive with an nth order reaction [24]. The material starts to degrade from a virgin state to a (degraded) final state (composed of carbonaceous residue and carbon fibre). So, the decomposition of the material is considered to be a multi-species decomposition (*α_1_* and *α_2_*) as given in Table 1. With the assumption of the constant volume, the density rate, *∂ρ/∂t* (with *t*, the time) can be expressed as a function of the kinetic decomposition model of each *i* steps.

### 3.2. Gas Mass Balance

The gas mass balance equation is expressed as a function of the density rate (Equation (1)). The accumulation of gases inside the material was neglected since no significant influence appears on the temperature profile of the material [11]. The gas storage is thus not taken into account in our model. A specific development was done in SAMCEF Amaryllis software in order to obtain gas mass transport vector, ${\dot{m}}_{g}^{\prime }$ in the three directions (*x,y,z*).

To take into account the internal pressure in the governing equation, Darcy’s law in three dimensions and the ideal gas law were used to link the pressure to the gas mass balance (Equations (2)–(5)).

(1) $$-\frac{\partial \rho }{\partial t}=\nabla \cdot \left[\begin{array}{c} {\dot{m}}_{g_{x}}^{\prime }\\ {\dot{m}}_{g_{y}}^{\prime }\\ {\dot{m}}_{g_{z}}^{\prime } \end{array}\right]$$

where,

(2) $$\left[\begin{array}{c} {\dot{m}}_{g_{x}}^{\prime }\\ {\dot{m}}_{g_{y}}^{\prime }\\ {\dot{m}}_{g_{z}}^{\prime } \end{array}\right]=\;-\frac{PM}{ℛT}\frac{\Gamma }{\mu }\cdot \;𝛻P$$

With

(3) $$\Gamma =\;\Gamma_{v}\frac{\phi_{\;}}{\phi_{v}}\;,$$

(4) $$\Phi =\left(1-\alpha \right)\phi_{v}+\alpha \phi_{e}\;$$

and

(5) $$\alpha =\frac{\rho_{v}-\rho }{\rho_{v}-\rho_{e}}$$

where *P* is the pressure, ***Γ***, the permeability tensor, *μ*, the dynamic viscosity, *ρ_g_*, the gas density, ***Γ_v_***, the virgin permeability tensor, *M*, the gas molecular mass, *R* is the universal gas constant, *Φ_v_*, the virgin porosity, *Φ_e_* , the final (end) porosity, and *Φ* , the porosity of the material, α, the decomposition degree, *ρ_v_*, is the virgin density of the material and *ρ_e_*, is the final density of the material.

In addition, the value of the virgin permeability tensor comes from the literature [27], since the measurement of the permeability in the 3D direction is a complicated task. An indirect measurement can be performed using an inverse method on the tomographic results but this would be time consuming, and he above assumption is sufficient [5,11]. As previously mentioned, the major issue with using more complicated models is the adequacy of available data to use as input [28].

### 3.3. Heat Balance

For the heat balance equation (Equation (6)), the heat transfer (I), the anisotropic heat conduction (II), the decomposition of the T700/M21 composite (III) and the gas transport linked to the internal pressure (IV) are considered. The accumulation of heat in the gas is neglected compared to the accumulation of heat in the solid.

(6) $$\underset{I}{\underset{︸}{\left[{\rho C}_{p}\right]\frac{\partial T}{\partial t}}}=\underset{II}{\underset{︸}{𝛻\cdot \left(\Lambda \;\cdot 𝛻T\right)}}\underset{\mathrm{III}}{\underset{︸}{\;-\;\left[{h-h}_{g}\right]\frac{\partial \rho }{\partial t}}}\underset{\mathrm{IV}}{\underset{︸}{-\left(\left[\begin{array}{c} {\dot{m}}_{g_{x}}^{\prime }\\ {\dot{m}}_{g_{y}}^{\prime }\\ {\dot{m}}_{g_{z}}^{\prime } \end{array}\right]\cdot \;\nabla h_{g}\right)}}$$

where

(7) $$h_{g}=\int_{T_{0}}^{T}C_{p_{g}}dT$$

and

(8) $$h_{\;}=Q_{di}+\int_{T_{0}}^{T}C_{p}\;dT$$

where *T* is the temperature, subscript *g*, the gases, ***Λ*** the thermal conductivity tensor, *C_p_*, the specific heat capacity, *h*, the enthalpy and *Q_di_*, , the heat of decomposition of each *i* step. To implement the enthalpy of gases and solids (Equations (7) and (8)), the primitive of the specific heat capacity interpolations determined in the first part of the paper [24] is calculated. A law of mixture between the virgin state and final state as a function of the decomposition degree is used to express the total specific heat capacity as well as the thermal conductivity (Table 1).

### 3.4. Material Thermophysical Properties

The required input data were density, thermal conductivity tensor, specific heat capacity, kinetic decomposition model, specific heat of gases, and heats of decomposition necessary for the domain equation (Equation (6)). The temperature-dependant properties have been determined as a function of decomposition degree [24]. Models used to express properties are detailed in Table 1.

### 3.5. Boundary Conditions

To determine the boundary conditions and their respective unknown inputs, the measured rear face temperature of a titanium plate is compared to the numerical results. As discussed in a previous work [1], the heat flux measured is not uniform on the surface of the plate. The iso-heat flux curves formed a circular shape on the surface of the plate. Thus, two axial symmetries, (Oxy) and (Oxz) are used.

The actual net heat flux on the exposed surface of the coupon, *q"_S,0_* , is given by Equations (9) and (10) where *x = 0* in (0yz) corresponds to the exposed face, *q”_r_* is the radiant heat flux from the propane flame determined in a previous work [11], *T_fl_* is the gas flame temperature, *h_fl_*, the convective heat transfer coefficient between the flame and the material, *ε*, the emissivity of the material, *h_g_*, the gas enthalpy and *AEHC* is the average effective heat of combustion. The last terms (IV and V) are the two additional interactions at the boundary-layer gases. The term IV on the right hand side is the surface blowing flux due to the out-gassing (combustible gases or not) at the surface of the sample. This term accounts for the reduction in heat transfer due to the transpiration of gases from decomposition into the boundary layer [29]. In this work, it will be referred to as the out-gassing term.

(9) $$q_{S,\;0}^{\prime \prime }=\varepsilon q_{r}^{\prime \prime }-\sigma \varepsilon T_{\;}{}^{4}+h_{fl}\left(T_{fl}-T\right)-\underset{IV}{\underset{︸}{{\dot{m}}_{g_{x}}^{\prime }\cdot h_{g}}}+\underset{V}{\underset{︸}{{\dot{m}}_{g_{x}}^{\prime }\cdot AEHC}}$$

where

(10) $$\varepsilon =\left(1-\alpha \right)\varepsilon_{v}+\alpha \varepsilon_{e}$$

The last term (V) is a positive feedback due to the ignition of the combustible gases released from the decomposition near the surface of the composite [1]. Similar boundary conditions have already been expressed by considering a “heat loss due to gases flowing out from the pores into the surroundings” [30]. This term has also been used in the ablation model on composite [31]. Other authors expressed these interactions at the exposed face of the sample [20], considering that “the mass flux blowing off of the heated surface instantly burns with the surrounding air”. They deactivated the out-gassing term when the gas burnt at the surface of the material. This assumption cannot be used in our case because the authors consider all the decomposition gases combustibles.

Considering the inflammation of the combustible gases near the surface, an additional input (AEHC) has to be included and estimated. The measurement of the HRR and mass loss of the T700/M21 under the MLCC test [22] are used to determine this input. The formula given by the cone calorimeter standard (ISO 5660-1 [32]) is used and presented in Equation (11).

(11) $$AEHC=\;\frac{\sum_{t=t_{TTI}}^{t_{TTE}}HRR\;\times \;S\;\times \;∆t}{m_{TTE}-m_{TTI}}$$

where *S*, is the surface area and *Δt*, the sampling time interval. The calculation is performed over the flaming phase. *TTI* is time-to-ignition and *TTE* is time-to-end of flame.

After determining the boundary condition at the exposed surface, the boundary condition at the unexposed surface, *q"_S,L,_* is expressed as a function of the radiative and convective heat transfer with the surrounding air (Equation (12)).

(12) $$q_{S,\;L}^{\prime \prime }=h_{rear}\left(T_{a}-T\right)+\varepsilon \sigma \left(T_{a}{}^{4}-T{}^{4}\right)-{\dot{m}}_{g_{x}}^{\prime }\cdot h_{g}$$

*h_rear_* is determined using the natural convection formula at a pressure of 1 atm and a temperature of 22 °C for a vertical wall of 0.1 m height.

### 3.6. Numerical Details

For the finite element mesh, two axial symmetries were considered in the plans (Oxy) and (Oxz). Analyses were also realised on the same mesh of a complete plate before considering the results. These symmetries allow for a reduction in the number of elements in the study and the time of calculation (currently around 3h30—CPU time).

The spatial discretisation of the plate and the insulated plate (named Calsil) is realised with 3D solid elements. The elements are quadratic with numerous degrees of freedom by nodes (temperature, pressure, gas mass flow, and density). Schemes of the model are presented in Figure 2.

On the top of the plate (exposed surface), the total heat flux determined in the previous part takes into account the heat flux from the propane flame, the interactions due to the out-gassing and to the combustion of the combustible gases near the surface (Equation (9)). On the cold face of the plate, convection and radiation transfer with ambient and interaction due to the out-gassing are considered to be representative of the performed test. On each side of the plate, a radiative heat loss is considered (Figure 2). No gases escape from the edges of the coupon during the test (impact on 100 × 100 mm² on a 150 × 150 mm² plate).

Finally, the pressures and initial internal pressure at the cold and exposed face was recorded at 1 atm, and the initial temperature was measured at 30 °C.

## 4. Comparison between the Experimental and Numerical Results

The numerical results are compared to the measured data (temperature, mass loss) and post-fire testing analyses of the coupons (decomposition front) are done.

A comparison between the predicted and measured masses has been performed and presented in Figure 3.

A good agreement is obtained between the predicted and measured mass of the T700/M21 composite. A maximum error of 3% is obtained between both curves (Figure 3). The time-to-ignition (TTI) is roughly captured by the model. Indeed, the predicted TTI is equal to 40s instead of 25 s, as determined experimentally. Both values are in the same range of order. To better understand why the predictive mass is slightly overestimated compared to the measured mass, the temperature profile predictions are compared to the experimental data.

The temperature profiles of an UD T700/M21 composite at x = 1, 2, 3 and 4 mm from the impacted face are presented in Figure 4 and compared to the numerical results. A discussion on the experimental results was explained in a previous work [1], including the assessment of the fire-induced damage of the T700/M21 composite. To summarize, from the beginning of the test up to 20s, the first phenomena is the conductive effect governed by the heat flux of the flame and the thermal diffusivity of the virgin material. Then, the heating rate slows down since the degradation front affects the first plies of the material (t1) and since the production and migration of gases released from the decomposition begin. These phenomena contribute to reducing the temperature rises through the laminate. At times corresponding to 60s (t2) in Figure 4, the temperature near the fire exposed surface increases. This elevation is due to a higher intensity of the flame (interaction between the decomposition gases released from the material with the propane flame), which changes the flame heat flux and accelerates the decomposition process. Finally, the less prominent the thermal degradation is, the less the gases are produced and can burnt at the surface exposed to fire. The temperature of the composite tends towards stabilisation as a function of the test duration.

In terms of the numerical results, an excellent agreement of up to t1 (near 10–30 s) is observed between the predictions and measurements, owing to the high accuracy of the virgin inputs of T700/M21 implemented in the model and to the appropriate initial boundary conditions. Similarly, the temperature measured by the thermocouples placed at x = 1 and 2 mm are quite well predicted after 100 s and 150 s of test duration, respectively. For the thermocouple located at x = 3 mm, the prediction overestimates the measurement at around 100 °C. It might be assigned to the delamination phenomenon, but in our case, no significant delamination is shown since the material studied is a UD T700/M21 [1]. Each ply in a UD composite material is stacked in the same direction, decreasing the ply stresses between each one and decreasing the delamination effects. Therefore, this difference is not due to a lack of implementation of the delamination effect in the model. This discrepancy is rather explained by the overestimation of the flame heat flux between t1 and t2 reported in Figure 4. There is a lack of phenomena taken into account in boundary conditions as explained in the introduction section. This is discussed in the next paragraph. Moreover, the temperature measured at the rear face (x = L = 4 mm—Figure 4) is also overestimated due to the boundary condition at the exposed face and due to the lack of precision of the measurement. The temperature was measured using a pyrometer at the rear face of the composite with an emissivity being only estimated. The change of thermo-optical properties should be measured and taken into account in the model, which can be due to the modifications of material surface and/or the out-gassing. Consequently, the accuracy of the temperature measurement decreases.

In Figure 4, lines t1 and t2 correspond respectively to the beginning of the decomposition and to the beginning of the inflammation [1]. The change of heating rates is not captured by the model. These discrepancies could come from a lack of accuracy of the input data of the thermochemical model, from the boundary conditions, or from both. As the TTI is only roughly captured by the model (Figure 3), its delay influences the temperature profiles. This induces a temperature deviation between the experimental and numerical results that increase with the increase of distance from the impacted face. To show why this is important, the beginning of the decomposition and a comparison between the numerical results of the pure conductive model and the full model with the experimental temperature at 3mm is presented in Figure 5.

The curves are well superimposed at the beginning of the temperature profile showing that the conduction governs the early stages of the tests. Then, differences between the predicted temperatures and the experimental ones are observed up to 250 °C for the pure conductive model, compared to only 85 °C for the full model. A reduction up to 165 °C is noticed using the current model instead of a pure conductive model that clearly evidences the importance of taking into account all the phenomena considered in the full model. However, the change of heating rates is not captured by the model at the right time. Just after the predicted TTI (40 s) with the full model, the fire behaviour of the T700/M21 creates a drastically change of the heating rate. The comparison suggests that if the prediction of the TTI is improved, the model can be improved. In addition, if the boundary condition from the propane flame is optimised, the prediction of the temperature profile is enhanced.

Furthermore, some inputs cannot be responsible for the overestimated temperature. Indeed, the first 30s was predicted by the model and, at 400 s – t3, the cooling rate of the temperature profiles is captured by the predicted results. These results validate the numerical implementation of the final emissivity as well as the final thermal properties (material totally degraded as shown on the tomographic image [1]) and the boundary conditions without interactions. It should be remembered that these interactions play a role in the boundary conditions at the exposed and rear face as long as there is out-gassing (Equations (9) and (12)). Even if uncertainties of the inputs influence the thermal response of the T700/M21 exposed to fire, they could be responsible for small discrepancies but not as much as observed in Figure 4. Indeed, the MLCC modelling case proved that when the inputs and the boundary conditions (without interactions) are well determined and known, the model accurately predicts the thermal response and mass loss of the T700/M21 [11]. Moreover, the influence of these interactions, i.e., positive feedback and out-gassing, in the previous model (MLCC) is not as important as the fire modelling case since the main difference between both modelling cases is (i) the incident heat flux (50 kW/m² vs. 116 kW/m²), (ii) a propane flame which can be interacted with the combustible gases released from the decomposition of the composite, and that (iii) the MLCC boundary conditions are better controlled compared to this fire test. In our experiment, the boundary conditions of the titanium plate have been verified without interactions. It makes sense that these discrepancies are mainly due to the determination of the boundary conditions: (i) a simplified formulation of the incident heat flux from the propane flame has been used and (ii) the changes of the incident heat flux from the propane flame, created by the interactions at the boundary-layer gases, are empirically taken into account.

It can be concluded that the overestimation of the predicted temperature profiles is due to a lack of certainty of the flame heat flux. Determining the heat flux at the exposed surface is still quite difficult without modelling the flame using CFD models, for example. More investigations must be performed on this topic.

Even if the temperature profiles are predicted quite well (as a result of the mass loss of the T700/M21 being slightly overestimated), the comparison between the numerical and observed front of decomposition can be discussed. Images of the coupons after 420 s of test duration and the calculation of the decomposition degree are compared in Figure 6.

It can be clearly observed that the material is degraded at the exposed surface in Figure 6a and slightly degraded under the insulated plate. The front of the decomposition follows the thermal conductive heat transfer of the UD T700/M21 (c.f. thermal conductivity tensor [24]). The same observation can be made on the numerical results (Figure 6b). In addition, the numerical results provide information on the front of decomposition which is more important on the border of the 100x100mm² exposed surface (red part). Moreover, a similar behaviour can be observed between the images and numerical results (Figure 6c,d). The front of decomposition is not uniform through the thickness of the material (Figure 6c)). Indeed, it is less important at the rear face of the sample, as shown in the numerical results (Figure 6d)).

Finally, Figure 6e shows the non-symmetric behaviour of the UD T700/M21 when exposed to fire. Therefore, even if the mass and temperature profile is slightly overestimated, the final state of the UD T700/M21 is predicted by the 3D thermochemical model.

## 5. Conclusions

A thermophysical model has been developed to simulate a novel fire test. The comparison between the experimental and numerical results reveals the capability of the model to predict the behaviour of the material. Two strong points are highlighted. The first one concerns the delamination phenomenon. It has been demonstrated that the lack of implementation of the delamination phenomena in the models is not necessary responsible for the lack of accuracy of numerical predictions. The predicted time-to-ignition and the implementation in the model of the boundary condition at the exposed face have to be improved. Another point concerns the unsatisfying determination of the heat flux at the exposed surface. In the case of direct fire impact, we highlighted the limits of the model due to the determination of the flame heat flux. The heat flux at the exposed face is overestimated, which causes an overestimation of the temperature profiles at the beginning of the decomposition. Thus, the determination of the flame boundary condition has to be revisited using, for example, a strong coupling between the current thermochemical model and a CFD approach.

This model that has been developed for predicting the thermochemical behaviour of a composite in fire is a dramatic enhancement compared to the previous literature models since (i) a competitive multi-step decomposition kinetic is included, (ii) all temperature-dependant inputs are determined experimentally up to 1000 °C and as a function of the decomposition degree, and (iii) near-surface empirical interactions between the composite laminate and the gas released from the decomposition are taken into account in a 3D thermochemical model. It is the first time that a 3D pyrolysis model is compared to experimental results when a carbon fibre/epoxy composite is exposed to fire (direct fire impact) given all input data necessary for the modelling, which are determined experimentally as a function of the decomposition degree and up to a high temperature (1000 °C). Therefore, it would be helpful to develop a new numerical model for fire safety engineering.

## Figures and Tables

**Figure 1:** Picture (**a**) and scheme (**b**) of the novel test bench [1].

**Figure 2:** Scheme in plane (Oyz) and with applied boundary conditions in plane (Oxy).

**Figure 3:** Comparison between the predicted and measured remaining mass.

**Figure 4:** Comparison of the experimental and numerical results of the temperature profile of the UD T700/M21 in fire.

**Figure 5:** Comparison between the measured temperature at x = 3 mm with the predicted temperature using a pure conductive and the current models.

**Figure 6:** Comparison of the damage front of the UD T700/M21 composite at the end of the fire test (420 s) between (**a**) the sample at exposed face; (**b**) the Samcef results the exposed face; (**c**) the section A-A of the sample; (**d**) the Samcef results at the section A-A and; (**e**) the Samcef results visually observed in 3D.

**Table 1:** Expression of thermophysical properties used in the three-dimensional thermochemical model.

Name	Unit	Model Used
Density, *ρ*	[kg/m^3^]	$\rho =\rho_{v}-\overset{2}{\underset{i=1}{\sum }}\Delta \rho^{i}\alpha_{i}$
		With
		$\{\begin{array}{c} \Delta \rho^{1}=Fraction1.\left(\rho_{v}-\rho_{e}\right)\\ \Delta \rho^{2}=Fraction2.\left(\rho_{v}-\rho_{e}\right) \end{array}$
Specific heat capacity, *C_p_*	[J/kg·K]	$C_{p}=\left(1-\alpha \right)C_{p_{v}}+\alpha C_{p_{e}}$
Thermal conductivity tensor, ***Λ***	[W/m·K]	$\Lambda =\left(1-\alpha \right)\Lambda_{v}+\alpha \Lambda_{e}$
Mass loss rate, *∂ρ/∂t*	[1/s]	$\{\begin{array}{c} \frac{\partial \alpha_{1}}{\partial t}=A_{1}{\left(1-\alpha_{1}-\alpha_{2}\right)}^{n_{1}}exp\left(\frac{-E_{a_{1}}}{ℛT}\right)\\ \frac{\partial \alpha_{2}}{\partial t}=A_{2}{\left(1-\alpha_{1}-\alpha_{2}\right)}^{n_{2}}exp\left(\frac{-E_{a_{2}}}{ℛT}\right)\left(1+Kcat.\alpha_{2}\right) \end{array}$
